# Pharmacological Potential of *Avicennia alba* Leaf Extract: An Experimental Analysis Focusing on Antidiabetic, Anti-inflammatory, Analgesic, and Antidiarrheal Activity

**DOI:** 10.1155/2022/7624189

**Published:** 2022-05-06

**Authors:** Saikat Mitra, Fahadul Islam, Rajib Das, Humaira Urmee, Aklima Akter, Abubakr M. Idris, Mayeen Uddin Khandaker, Mohannad A. Almikhlafi, Rohit Sharma, Talha Bin Emran

**Affiliations:** ^1^Department of Pharmacy, Faculty of Pharmacy, University of Dhaka, Dhaka 1000, Bangladesh; ^2^Department of Pharmacy, Faculty of Allied Health Sciences, Daffodil International University, Dhaka 1207, Bangladesh; ^3^Department of Pharmaceutical Science, North South University, Dhaka 1229, Bangladesh; ^4^Department of Chemistry, College of Science, King Khalid University, Abha 62529, Saudi Arabia; ^5^Research Center for Advanced Materials Science (RCAMS), King Khalid University, Abha 62529, Saudi Arabia; ^6^Centre for Applied Physics and Radiation Technologies, School of Engineering and Technology, Sunway University, Bandar Sunway, Petaling Jaya 47500, Malaysia; ^7^Department of Pharmacology and Toxicology, Collage of Pharmacy, Taibah University, Madinah 41477, Saudi Arabia; ^8^Department of Rasa Shastra and Bhaishajya Kalpana, Faculty of Ayurveda, Institute of Medical Sciences, Banaras Hindu University, Varanasi, 221005 Uttar Pradesh, India; ^9^Department of Pharmacy, BGC Trust University Bangladesh, Chittagong 4381, Bangladesh

## Abstract

*Avicennia alba* is a mangrove plant that is extensively used to treat severe health issues. This focus of this study was to investigate the antidiabetic, anti-inflammatory, analgesic, and antidiarrheal activities of methanolic extract of *A. alba* leaves in Swiss albino mouse model. The antidiabetic, anti-inflammatory, analgesic, and antidiarrheal activities of the leaf extract were performed using alloxan-monohydrate, carrageenan-induced paw edema, acetic acid-induced writhing test and the hot plate method, and castor oil-induced method, respectively. The extract was used at doses ranging from 200 to 500 mg/kg to conduct the investigation. Leaf extract at 400 and 500 mg/kg showed potent antidiabetic activity in alloxan-induced diabetic mice. Advanced research is needed to control blood glucose levels and carrageenan paw edema-based anti-inflammatory effects. Both tests showed statistically significant result in a dose-dependent manner. The maximum dose (500 mg/kg) demonstrated potent analgesic activity in both writhing test and hot plate method. The plant extract also showed significant antidiarrheal activity at 400 and 500 mg/kg in experimental mice. However, more research is needed to explore the possible mechanisms and isolate the compounds associated with these bioactivities from the leaf extract of *A. alba*.

## 1. Introduction

Medicinal plants produced in mangroves are commonly used to treat many severe maladies [1–3]. *Avicennia alba* is a mangrove plant that belongs to the Acanthaceae family and referred to as “Ilva mada.” It grows in tropical regions and found far from the ocean [4]. The reason behind of its name was two Latin phrases “Alba” and “putih,” which indicate “white” in Latin and Malay, respectively. It is more ubiquitous on near about the rivers or on freshly formed mudbanks on the seaward side. In some ways, it is a precursor to animals that can survive in a protected environment. *A. alba*'s leaves and fruit morphologies can be “abnormal” if the tree is growing in the shade or suffering from low nutrition or other difficult circumstances. Normally, the flowers are little and golden, and they are usually spread out across an area. There is a long, tapering pointed end to the fruit, which is teardrop-shaped [5, 6]. Together with nutrition and fiber, the phytochemicals from *A. alba* provide a widespread defensive function against physiological complications and stress conditions. The most abundant bioactive compounds include carbohydrates, tannins, alkaloids, flavonoids, terpenoids, steroids, and phenolic compounds [7–9].

The leaves of *A. alba* were tested for antioxidant activity and appeared to be effective [10–12]. In traditional Chinese medicine, the bark and seeds of *A. alba*'s were employed as a fish poison, while the resin was used to treat birth control, ulcers, skin conditions, and even cancer [13]. *A. alba*, a mangrove, has been subjected in very few studies. Its crude extract has been shown to be effective against polymicrobial diseases [14]. *A. alba* leaves protect gastric mucosa from ethanol-induced damage [15], and the stem of the plant has been used to isolate and structurally elucidate new naphthoquinones and their analogues [1, 6]. Plant and human pathogenic bacteria, particularly oral pathogens, were shown to be inhibited by *A. alba* [13, 14]. Additionally, the plant extract has antifungal properties. Aphrodisiacs, skin disease, asthma, rheumatism, scabies, antifertility agents, paralysis, snake bites, and ulcers are only some of the conditions for which *A. alba* is employed in the Indian medical system [7, 16].

Diabetes is a common chronic disease, characterized by recurrent hyperglycemia and metabolic problems [17]. Diabetes mellitus (DM) is the eighth major cause of death, affecting 4% of world population. Its effect on various physiological systems, especially nerves and blood flow, makes it a severe medical condition in both developing and industrialized countries [18, 19]. Despite claims by trado-medical practitioners that they have a treatment for DM, there is no cure. It falls into the same category as AIDS, cancer [20, 21], and hypertension, which can only be controlled at the moment [22–24].

Inflammation is triggered due to numerous unpleasant stimuli including pathogens and physical trauma, which is used by immunological responses [25, 26]. Conversely, pain is regarded as a negative sensory and emotional perception linked to tissue injury. It is also frequently triggered by unpleasant stimulus and conveyed to the central nervous system (CNS) via specific neural networks, where it is recognized [27, 28]. It is a strategy of safeguarding the body from damage. Despite the development of sufficient medications, inflammation and pain continue to be the difficult and debilitating health issues, affecting 80% of the adult population worldwide [29]. Untreated and chronically protracted pain is the most common ailment, causing both harm and injury. Nonresolving inflammation also causes functional impairment, such as taking time off work, school, or community engagements, and can lead to the development of serious inflammatory conditions such as asthma, autoimmune disorder, systemic inflammatory, glomerulonephritis, inflammatory bowel disease, and rheumatoid arthritis [30, 31]. These debilitating diseases are the leading cause of disability and, if not appropriately monitored and maintained, can lead to death. Standard pain and inflammation medications are still the backbone for treating and managing these conditions [32]. However, they are concomitant to various health consequences and toxicity, including stomach irritation, gastric ulcer, alteration kidney function, hypertension implications, liver damage, and platelet suppression, which can lead to increased bleeding [33, 34].

Diarrhea is of major concern for morbidity and mortalities in third world nations, affecting primarily neonates and infants [35, 36]. As per UNICEF and WHO data, yearly 2.5 billion cases of diarrhea are reported worldwide; with 1.9 million children under the age of five dying from diarrhea, the majority are from developing nations. 78% of diarrheal deaths of children occur in Africa and Southeast Asia [37, 38]. Antimotility and antisecretory medications are the mainstays of diarrhea management. Opioids and their metabolites are still commonly utilized to treat diarrhea. Opioid antidiarrheals such as diphenoxylate, difenoxin, and loperamide are routinely utilized [39]. Several alternative medications that have antimotility or antisecretory properties on the bowel and can be used to treat diarrhea exist [40].

Therefore, there is a compelling necessity expand research into phytochemicals that are useful to relieve pain and inflammation. The purpose of the study is to evaluate pharmacological activity of *A. alba*, focusing on antidiabetic, anti-inflammatory, analgesic, and antidiarrheal activities in Swiss albino mouse model.

## 2. Materials and Methods

### 2.1. Chemicals and Plant Material

The standard drugs glibenclamide, indomethacin, diclofenac sodium, morphine, and loperamide were purchased from Incepta Pharmaceuticals Ltd., Dhaka, Bangladesh. Different reagents and distilled water were also purchased from British Drug House (BDH) Chemicals Ltd., Dhaka, Bangladesh. Plant material from *A. alba* was collected from Sylhet. The plant's genus and family were reported from National Herbarium, Bangladesh (DACB accession number: 40556).

### 2.2. Preparation of Methanol Extract

The *A. alba* leaves were harvested and cleaned with distilled water for the removal of undesirable materials. First, leaves were sun-dried before being processed into a coarse powder. Before the study began, container was used to place the powder into it and kept in a dry, cool, and dark setting. In a glass flask, 400 gm of granulated leaves of *A. alba* was steeped for 10 days in 1000 ml of 95% methanol with constant shaking and mixing. To get a clean filtrate, filtration was done for the entire mix via a fine and white cotton material and Whatman filter paper No. 1. The filtrate was kept in an open room to disperse the solvent, and the extract was found. The methanol extract of the leaves yielded 2.11% *w*/*w* yield. Extract was redissolved in 5% DMSO for oral administration.

### 2.3. Experimental Animals

Swiss albino mice (*n* = 90) of both sexes (20-25 g) were procured from Jahangirnagar University in Dhaka, Bangladesh, and maintained in animal cages under regular natural circumstances (22-25°C, moistness 60-70%, 12-hour light: 12-hour dull cycle). A regular pellet fed was fed to the mice. The Faculty of Allied Health Sciences Research Ethics Committee, Daffodil International University, Dhaka-1207, Bangladesh, accepted all of the procedures used in this investigation, including the use of animals (Ref: FAHSREC/DIU/2020/1006).

### 2.4. Phytochemical Group Screening

In the preliminary phytochemical study, the presence of certain phytochemical groups was evaluated. Colorimetric methods were used to identify flavonoids, saponins, tannins, carbohydrates, alkaloids, terpenoids, gums, phenolics, steroids, and glycosides [41–43].

### 2.5. Acute Toxicity Test

The extract was administered to mice in oral route (*n* = 5) at doses of 100, 200, 400, and 600 mg/kg, with % mortality measured from 24 to 7 days [44, 45].

### 2.6. Antidiabetic Activity

#### 2.6.1. Experimental Design

Into five groups, the mice were separated, five mice per group. Group I was a standard control (saline, nondiabetic), group II was alloxan- (150 mg/kg-) treated control (diabetic control), group III was provided glibenclamide (10 mg/kg), and groups IV, V, and VI were taken leaf extract at doses of 200, 400, and 500 mg/kg, respectively. For 15 days, the therapeutic options were continued. The extracts and saline solution were administered orally administered.

The extract was used to evaluate the antidiabetic activity using albino mice at 200, 400, and 500 mg/kg b.w. doses in an oral glucose tolerance test in vivo. The doses were designated on the basis of their efficacy in previous studies [44].

#### 2.6.2. Blood Glucose Determination

A fractional tail amputation process was used to detect each mouse's blood glucose level, and blood was drawn from the tail vein using a one-touch electronic glucometer with glucose test strips. The tails were rinsed in ethanol to prevent them from infection [46].

#### 2.6.3. Body Weight (b.w.) Analysis

The experimental mice bodyweight is measured before they began the medication (day 0) and throughout the trial (days 7 and 15), as well as fluctuations in weight.

### 2.7. Anti-inflammatory Activity by Carrageenan-Induced Inflammatory Method

The animals were separated into 5 groups of fine mice each on the day of the experiment. They were weighted to ensure that the medication was administered correctly. Group I received 1% Tween, while groups III, IV, and V provided leaf extract at 200, 400, and 500 mg/kg b.w. doses. In group II, any anti-inflammatory medicine might be employed as a positive control. Indomethacin was utilized as the standard in this model. The animals were given 0.1 ml of 1% carrageenan in the subplanter region of the right hind paw after 30 minutes. At the level of the lateral alveolus, the paw was tagged with a permanent marker. A plethysmograph was used to take the initial reading right after the injection, as well as successive paw volumes. Paw volumes were measured at 0, 30, 60, and 120 hours. Afterward, carrageenan was injected. The volume of edema was estimated by subtracting the initial volume from the volume of the time points in consideration [47].

### 2.8. Analgesic Activity Test

#### 2.8.1. Acetic Acid-Induced Abdominal Writhing Test

The experiment for analgesic activity proceeded with categorizing the mice into 5 groups. Each mice group contains 5 mice, standard (10 mg/kg diclofenac sodium in intraperitoneal route) and control (0.5% methylcellulose). Groups III, IV, and V were considered with methanol extract of *A. alba* leaves at dosages of 200, 400, and 500 mg/kg b.w., respectively. Writhing assay was followed for the assessment of analgesic activity induced by acetic acid. For the following 10 min after obtaining test data and vehicle orally 30 minutes before intraperitoneal delivery of 10 ml/kg of 0.7% acetic acid, the mice were examined for particular body contraction known as “writhing” [7]. Fifteen minutes prior to the acetic acid injection, diclofenac-sodium was given intraperitoneal injection. The percent of protective action against writhing induced by acetic acid was calculated using the formula.

(1) $$\begin{array}{c} \text{Percentage protection}=\frac{\left(Wc-Wt\right)}{Wc}\times 100, \end{array}$$

where *Wc* and *Wt* are the mean values of the control and treated groups, respectively.

#### 2.8.2. Hot Plate Test

This test was performed as per the instructions provided by previous researchers [48]. Methanol leaf extract (200, 400, and 500 mg/kg b.w. p.o.), morphine (5 mg/kg b.w. p.o.), and normal saline (10 ml/kg b.w.) were introduced orally to 5 mice groups (*n* = 5). Mice were kept on a hot plate (Bibby Sterilin, UK), and the latency of reaction (in seconds) for licking the jumping or hind paw was measured. The mice for the studies were those that reacted within 15 seconds and did not exhibit a lot of variance. Before and after treatment with the various medicines, recordings were collected at 0, 30, 60, 90, and 120 mins [49].

### 2.9. Castor Oil-Induced Antidiarrheal Activity Test

This experiment was proceeded as per the instructions of Islam et al. [50]. Before the test, the animals were separated for the diarrheal test by introducing them castor oil (0.5 ml) in oral route, and then, animals with diarrheal symptoms were selected for experimental purpose. Five groups were divided with 25 mice (five in each group). Before going through the experiment, mice were starved for 18 hours (only water was accessible). Animals in group I were given merely the vehicle (1% Tween 80, 10 ml/kg, i.p.) as a control, while those in group II were given the conventional medicine (loperamide 3 mg/kg b.w.). The extract doses for groups III, IV, and V were 200, 400, and 500 mg/kg, respectively. Castor oil (0.5 ml) was introduced to mice in oral route 30 min afterward treatment to tempt diarrhea and were individually placed in blotting paper. The paper was replaced every hour. Diarrheal feces were counted, and the proportion of defecation inhibition was computed for each group over a 4-hour observation period.

### 2.10. Statistical Analysis

The SPSS (Statistical Package for the Social Sciences) statistical software, version 20.0, was used for all the data analysis. The results are demonstrated as the mean ± SEM (standard error mean) value. The statistical analysis was accomplished using one-way analysis of variance (ANOVA) pursued by Dunnett's test for all the experiments. ∗*P* < 0.05, ∗∗*P* < 0.01, and ∗∗∗*P* < 0.001 were reported to be statistically significant.

## 3. Results

### 3.1. Phytochemical Screening

Phytochemical investigation on the methanol leaf extract of *A. alba* demonstrated the occurrence of flavonoids, saponins, tannins, alkaloids, terpenoids, gums, phenolics, carbohydrates, and steroids, as well as the absence of glycosides (Table 1).

### 3.2. Acute Toxicity

Normal behavior was observed in mice given the extract at doses of 100–600 mg/kg p.o. They were awake and alert, with typical grooming, contact, and pain responses. Passivity, stereotypy, or vocalization was not present. They had typical motor activity and secretory indications. The animal's alertness, grip strength, limb tone, motor activity, and gait were all normal. In mice, the extract was determined to be safe up to 600 mg/kg.

### 3.3. Antidiabetic Activity

#### 3.3.1. Blood Glucose Level

The leaf extract of *A. alba* given at 200, 400, and 500 mg/kg reduced glucose levels of blood in diabetic mice dose dependently at the end of the trial, although not as much as glibenclamide-treated mice (Table 2).

#### 3.3.2. Body Weight Changes and Fasting Blood Glucose Levels

In alloxanized diabetic mice, the leaf extract at dosages of 200, 400, and 500 significantly increased b.w. and generated a maximum drop in fasting glucose levels after 15 days of therapy (Table 3).

### 3.4. Anti-inflammatory Activity

The methanol extract of *A. alba* demonstrated to have anti-inflammatory activity in mice at dose levels of 200, 400, and 500 mg/kg/day b.w., respectively. Indomethacin (10 mg/kg) for leaf was found to have anti-inflammatory activity in mice at dose level of 500 mg/kg/day body weight, respectively (Table 4).

### 3.5. Analgesic Activity

#### 3.5.1. Writhing Test

Methanol leaf extract of *A. alba* inhibited writhing by 39.01, 56.74, and 64.18% at dosages of 200, 400, and 500 mg/kg b.w., respectively, whereas diclofenac sodium repressed writhing by 69.86% at a dose of 10 mg/kg, and the findings were statistically significant (∗∗*P* < 0.01, ∗∗∗*P* < 0.001) (Table 5).

#### 3.5.2. Hot Plate Test

At 90 min, the leaf extract of *A. alba* revealed maximum reaction times of 7.24, 8.40, and 9.10 seconds for dosages of 200, 400, and 500 mg/kg, respectively, whereas morphine demonstrated a maximum reaction time of 11.01 sec for dosages of 5 mg/kg at 90 min (Table 6). The findings showed that the extract considerably improved (∗*P* < 0.05, ∗∗*P* < 0.01) pain threshold when comparison was done to the control group, and that the effect lasted for the full 120-minute monitoring period.

### 3.6. Castor Oil-Induced Antidiarrheal Activity

At dosages of 200, 400, and 500 mg/kg, the three serial dosages of *A. alba* leaf extract effectively reduced enterpooling in mice induced by castor oil. The largest dosages of leaf extract (400 and 500 mg/kg) lead to a greater diminution in both the total amount of diarrheal feces and percent inhibition of diarrhea. When compared to the negative controls, the leaves extract inhibited diarrhea by 30.91% and 46.36% at 400 and 500 mg/kg dosages, respectively. Loperamide had the highest percent inhibition of diarrhea, at 59.09% (Table 7).

## 4. Discussion

Many traditional medicines rely heavily on the medicinal properties of plants [51, 52]. There may be polar plant elements in *A. alba* since it grows in coastal woods. Methanol was employed in this experiment. The solvent was entirely evaporated to dryness in order to prevent any influence on the experimental animals [53]. There is a long history of therapeutic usage of the herb studied in this research, both in India and elsewhere [16]. *A. alba* leaf extract was analyzed for phytochemicals, and the results are reported in Table 1. The methanol extract of *A. alba* leaves displayed the occurrence of saponins, flavonoids, tannins, sugars, alkaloids, terpenoids, gums, phenolics, steroids, and the lack of glycosides. Leaf extract in methanol had more phytochemicals than the other extracts studied. Most secondary metabolite adaptive value remained undiscovered for many years. Metabolic wastes, it was assumed, were the only sources of these chemicals. Today, we know that a large number of secondary metabolites in plants have ecological roles. The research demonstrates that *A. alba* is an extremely diversified phytochemically. Thus, these phytochemicals have a dramatic effect on plants' capacity to compete and adapt. The study of these chemicals is fascinating because they may be useful as pharmaceuticals, poisons, flavors, and industrial materials. Numerous polyphenolic chemicals found in mangrove plants, including as tannins and flavonoids, were documented to possess a variety of pharmacological properties, including antidiarrheal and analgesic properties. Plant flavonoids and pentacyclic triterpenes may act as an analgesic in rats [54]. Additionally, this research discovered that benzoquinones may block lipoxygenase pathway, which supports the usage of *A. alba* in traditional medicine to treat diarrhea. Tannins and saponins are also present and contribute to the antidiarrheal activity. Ahmed et al. [53] shown that the occurrence of alkaloids, steroids, and glycosides in the leaves of *A. alba* may result in analgesic and antidiarrheal activity.

Using a writhing model induced by acetic acid in mice, the methanol extract of *A. alba* was shown to have analgesic properties. Models of pain feeling are generated by inducing localized inflammation in response to acetic acid injections. The algesia caused by the release of endogenous chemicals by acetic acid, which is employed to produce writhing, excites the pain nerve endings [55]. It was suggested that acetic acid when injected intraperitoneally causes pain because of elevated PGF2 and PGE2 levels [56]. The extract had equivalent writhing inhibition to diclofenac sodium, the usual medication (Table 5). The analgesic properties of the extract are because of the polar molecules. This finding suggests that *A. alba*'s methanol extract may have analgesic properties. Radiating heat is also used to investigate central and peripheral effects. Thus, the findings are corroborated by the plant's ability to inhibit both peripheral and central pain pathways by the use of methanol extract. The development of heat discomfort is associated with two kinds of sensory neurons in the skin: delta and C fibers. Additionally, the skin has a high concentration of temperature-sensitive ion channels. Calcium and sodium ions can pass through the plasma membrane because it has transmembrane proteins that let them do so. In order to pinpoint the cause of pain, the brain processes action potentials generated by the ions and sends them to the spinal cord. Heat-inducing discomfort may be alleviated by analgesic herbs' ability to modulate signal conduction and action potential [57].

A diarrhea model induced by castor oil in mice was utilized to test the *A. alba* extract's antidiarrheal activity. There are several theories explaining castor oil's diarrheal impact, including the blockage of Na^+^, K^+^-ATPase activity, adenylate cyclase activation, or the commencement of prostaglandin (PG) production, PAF (paroxysmal atrial fibrillation), and nitric oxide (NO). When mixed with bile and pancreatic enzymes, castor oil causes diarrhea and releases ricinoleic acid from triglycerides when taken orally. The colon is the primary site of absorption and excretion of ricinoleic acid and has influence on absorption or secretion. The ricinoleate salts with K^+^ and Na^+^ quickly develop in the lumen of the gut as a result of the liberation of ricinoleic acid. It acts like a soap or surfactant on the mucosal surface of the digestive tract and in the intestines itself. As a general rule, ricinoleate salts induce adenyl cyclase [58] or the release of PG in intestinal epithelial cells [59]. The extract lowered the frequency of defecation and the total stool count while increasing the latent period. In addition, the *A. alba* extract contains flavonoids that have been shown to suppress the production of autacoids and prostaglandins, which means that castor oil's effects on motility and secretion may be inhibited. Antidiarrheal properties of this extract may potentially be attributable to the formation of protein tannates, which in turn strengthen the intestinal mucosa and limit secretion [60].

Antidiabetic activity as measured by body weight and fasting blood glucose level is shown in Tables 2 and 3. In disease control rats, body weight is observed to be dramatically lowered when compared to normal control rats. The therapy with a specific herbal extract resulted in a rise in body weight. Increased body weight indicates that certain herbal extract dosages have an antihyperglycemic effect. In fasting blood glucose tests, alloxan-induced diabetic rats had an increased level of glycated hemoglobin (HbA1c) owing to an increase in blood glucose levels, which react with hemoglobin and result in the creation of glycated hemoglobin [61, 62]. The methanol extracts dramatically decreased blood glucose levels, which resulted in a drop in glycosylated hemoglobin levels. When compared to other treatment groups, the high dosage (400 and 500 mg/kg) of methanol extract *A. alba* shown superior potency. The term “fat vacuoles” or “steatosis” refers to the intracytoplasmic accumulation of triglyceride (neutral fats) in the liver of rats after alloxan injection. Accumulation of these neutral fats in the liver resulted in nonalcoholic fatty liver disease (NAFLD), which is described by hepatocyte fatty alterations, ballooning degeneration, mixed lobular inflammation, and fibrosis. Ballooning is the most significant aberration in NAFLD because it results from hepatocytes losing their usual polygonal shape and becoming bloated and spherical because of intracellular fluid buildup initiated by microtubule malfunction and decreased protein secretion [61]. Hepatic fibrosis occurs when stellate cells in the liver progressively lose their ability to produce collagen. High dosages of methanol extract from *A. alba* showed improved hepatoprotective action and preservation of the normal liver architecture, respectively [63].

It is demonstrated in this research that methanol extract of *A. alba* does not induce acute toxicity, since the LD50 value exceeds 600 mg/kg. There were no deaths or evidence of toxicity in mice treated with extracts at a level of 600 mg/kg, proving their safety in usage. Additionally, it was shown to be as safe when used in an erythrocyte hemolytic experiment [63]. For this reason, methanol *A. alba* extracts may be employed as a safe phytochemical to treat various maladies. Inflammation is caused by the breakdown of proteins, which is well-documented. Anti-inflammatory medications such as salicylic acid, phenylbutazone, and flufenamic acid, among others, have shown dose-dependent capacity to denaturate thermally generated proteins. Anti-inflammatory efficacy was tested as a means to determine the extract's potential to suppress protein cleavage. According to Mondal et al. [64], methanol extract of *A. alba* was efficient in preventing heat-induced albumin denaturation at various doses. The in vitro anti-inflammatory effect of the studied ethanol extract was also shown to be promising. When living tissues are injured, they respond by inflaming themselves. It is a multistep process that includes mediator release, enzyme activation, fluid extravasation, tissue breakdown, cell migration, and repair [64]. Carrageenan-induced acute inflammation in rats was shown to be significantly reduced by the methanol extract of *A. alba* in the current investigation [65]. A number of arachidonic acid metabolites, including prostaglandins, enhance the cardinal signs of inflammation; leukotriene B4 is a facilitator of leukocyte stimulation in the inflammatory cascade [64]. According to the findings, *A. alba* methanol extracts reduced carrageenan-induced rat paw edema at doses of 200 mg/kg, 400 mg/kg, and 500 mg/kg (Table 5). The suppression of some or all of the mediators produced within 90 hours following carrageenan injection is most likely the origin of anti-inflammatory effect against acute inflammation. NO is produced when PGs, cytokines, and iNOS are activated, indicating an inflammatory response [65]. Vasodilatation, an increase in vascular permeability, and the development of edema are all due to the action of NO. NO inhibition may be due to a mechanism that prevents iNOS activity and may also be responsible for the reduction of PG production. Finally, the data show that *A. alba* ethanol extract significantly reduces rat experimental inflammatory responses. According to past research, tannins, flavonoids, and phenolic chemicals in the plant may be responsible for this action. Therefore, further research is needed to identify the active chemical and determine if it may be used to treat chronic inflammation.

## 5. Conclusions

In conclusion, it was shown that the *A. alba* extract is a natural and harmless treatment with antidiabetic, anti-inflammatory, analgesic, and antidiarrheal action at doses up to 500 mg/kg. Our new results provide a scientific explanation for the plant's traditional usage. Remarkably, the methanol extract of *A. alba* displayed both central and peripheral analgesic activity, which might be attributable to the existence of such active components, since the herb has a long history of folk usage in pain and fever. Additionally, the research mentions *A. alba* leaf methanol extract's antidiabetic properties. The extract dosages (400 and 500 mg/kg) avoided excessive weight loss and maintained a favorable control of glycosylated hemoglobin. Finally, it is possible that the *A. alba* leaf has analgesic and antidiarrheal properties. These data support *A. alba*'s usage as a traditional medicine on a scientific foundation. However, further tests may be necessary to assess the plant's medicinal potential as a treatment.

## Figures and Tables

**Table 1:** Phytochemical screening of the leaf extract of *A. alba*.

Tested groups	Methanol leaf extract
Flavonoids	**+**
Saponins	**+**
Tannins	**+**
Carbohydrates	**+**
Alkaloids	**+**
Terpenoids	**+**
Gums	**+**
Phenolics	**+**
Steroids	**+**
Glycosides	-

(+) indicates presence; (-) indicates absence.

**Table 2:** The effect of *A. alba* leaf extract on alloxan-induced diabetic mice's blood glucose levels.

Group	Dose (mg/kg)	Blood glucose level (mg/dl)				
		Day 0	Day 4	Day 7	Day 10	Day 15
Normal saline	0.3 ml	122.60 ± 3.10	114.20 ± 1.07	108.10 ± 2.48	106.60 ± 2.70	98.8 ± 3.10
Diabetic control	0.3 ml	415 ± 4.50	423.15 ± 1.87	429.55 ± 3.10	438.10 ± 1.58	454.10 ± 3.20
Glibenclamide	10	394.20 ± 2.37	373.25 ± 2.31^∗^	339.15 ± 2.29^∗^	296.15 ± 3.06^∗∗^	265.27 ± 2.67^∗∗^
Methanol extract	200	401.30 ± 2.51	388.25 ± 2.27	372.55 ± 3.40	361.40 ± 3.24	344.25 ± 3.15^∗^
Methanol extract	400	385.25 ± 3.27	370.35 ± 2.57	360.30 ± 3.34^∗^	309.90 ± 3.14^∗∗^	285.10 ± 2.96^∗∗^
Methanol extract	500	387.55 ± 3.27	374.15 ± 3.24	366.45 ± 2.22	313.35 ± 3.27	291.25 ± 2.37

Results are expressed as mean ± SEM (*n* = 5), ^∗^*P* < 0.05, ^∗∗^*P* < 0.01, which considered significance compared with the control group (one-way ANOVA followed by Dunnett's test).

**Table 3:** The effects of *A. alba* extract on mice's body weight.

Group	Dose (mg/kg)	Body weight (g)				
		Day 0	Day 4	Day 7	Day 10	Day 15
Normal saline	0.3 ml	23.90 ± 0.27	25.14 ± 0.19	26.10 ± 0.18	27.20 ± 0.12	28.15 ± 0.21
Diabetic control	0.3 ml	27.20 ± 0.44	27.80 ± 0.17	25.55 ± 0.40	25.15 ± 0.22	24.10 ± 0.50
Glibenclamide	10	29.55 ± 0.22	30.25 ± 0.40	32.15 ± 0.25^∗^	33.65 ± 0.12^∗∗^	34.45 ± 0.10^∗∗^
Methanol extract	200	26.10 ± 0.25	26.10 ± 0.21	29.95 ± 0.35	30.85 ± 0.35	32.45 ± 0.20^∗^
Methanol extract	400	25.30 ± 0.15	26.25 ± 0.20	32.80 ± 0.14^∗^	32.25 ± 0.10^∗^	33.40 ± 0.45^∗∗^
Methanol extract	500	26.24 ± 0.11	26.50 ± 0.36	32.95 ± 0.42^∗^	32.85 ± 0.27^∗^	33.95 ± 0.23^∗∗^

Results are expressed as mean ± SEM (*n* = 5), ^∗^*P* < 0.05, ^∗∗^*P* < 0.01, which considered significance compared with the control group (one-way ANOVA followed by Dunnett's test).

**Table 4:** Appraisal of anti-inflammatory activity of *A. alba* leaf extract by carrageenan-induced inflammatory method.

Group	Dose (mg/kg)	Paw edema (mm)			
		0 hrs	30 hrs	60 hrs	90 hrs
Control	1% Tween	7.75	7.25	7.0	7.07
Indomethacin	10 mg/kg	4.29	4.22	3.75	3.71
Methanol extract	200	6.27	6.25	6.10	5.95
Methanol extract	400	5.88	5.77	5.60	5.50
Methanol extract	500	4.99	3.87	3.75	3.55

**Table 5:** Effect of leaf extract of *A. alba* using acetic acid-induced abdominal writhing test.

Group	Dose (mg/kg)	Writhing (mean ± SEM)	% of inhibition
Control	0.5% methylcellulose; 10 ml/kg	28.2 ± 0.89	—
Diclofenac sodium	10	8.5 ± 0.75	69.86^∗∗∗^
Methanol extract	200	17.2 ± 0.40	39.01^∗∗^
Methanol extract	400	12.2 ± 0.65	56.74^∗∗∗^
Methanol extract	500	10.10 ± 9.36	64.18^∗∗∗^

Results are demonstrated as mean ± SEM (*n* = 5), ^∗∗^*P* < 0.01, ^∗∗∗^*P* < 0.001, which considered significance compared with the control group (one-way ANOVA followed by Dunnett's test).

**Table 6:** Effect of leaf extract of *A. alba* using hot plate test.

Group	Dose (mg/kg)	Reaction time (sec)				
		0 min	30 min	60 min	90 min	120 min
Control	1% Tween 80, 10 ml/kg	4.07 ± 0.70	4.01 ± 0.37	4.0 ± 0.08	6.6 ± 0.40	4.15 ± 0.14
Morphine	5	4.10 ± 0.10	6.15 ± 0.16^∗^	8.50 ± 0.12^∗^	11.01 ± 0.18^∗∗^	9.60 ± 0.20^∗∗^
Methanol extract	200	4.19 ± 0.13	4.55 ± 0.22	5.55 ± 0.14	7.24 ± 0.20^∗∗^	6.40 ± 0.15^∗^
Methanol extract	400	4.44 ± 0.25	4.67 ± 0.37	6.44 ± 0.21^∗^	8.40 ± 0.15^∗∗^	6.80 ± 0.12^∗∗^
Methanol extract	500	4.55 ± 0.86	5.0 ± 0.14^∗^	6.90 ± 0.20^∗^	9.10 ± 0.31^∗∗^	7.0 ± 0.13^∗∗^

Results are expressed as mean ± SEM (*n* = 5), ^∗^*P* < 0.05, ^∗∗^*P* < 0.01, which considered significance compared with the control group (one-way ANOVA followed by Dunnett's test).

**Table 7:** Effects of leaf extract of *A. alba* in castor oil-induced antidiarrheal test.

Group	Dose (mg/kg)	Total number of feces (mean ± SEM)	% inhibition of defecation	Total number of diarrheal feces (mean ± SEM)	% inhibition of diarrhea
Control	1% Tween 80, 10 ml/kg	8.25 ± 0.50	—	5.50 ± 0.27	—
Loperamide	3	3.25 ± 0.23	60.61	2.25 ± 0.15	59.09
Methanol extract	200	6.10 ± 0.31	26.06	4.90 ± 0.34	10.91
Methanol extract	400	5.50 ± 0.15	33.33^∗^	3.80 ± 0.21	30.91^∗^
Methanol extract	500	4.90 ± 0.27	40.61^∗∗^	2.95 ± 0.19	46.36^∗∗^

Results are expressed as mean ± SEM (*n* = 5), ^∗^*P* < 0.05, ^∗∗^*P* < 0.01, which considered significance compared with the control group (one-way ANOVA followed by Dunnett's test).

## Data Availability

The data used to support the findings of this study are included within the article.
